The article "Segmentation and Automatic Identification of Vasculature in Coronary Angiograms" was published in 2021. Journal: Comput Math Methods Med.

# Segmentation and Automatic Identification of Vasculature in Coronary Angiograms

**DOI:** 10.1155/2021/2747274

**Published:** 2021-10-07

**Authors:** Yaofang Liu, Wenlong Wan, Xinyue Zhang, Shaoyu Liu, Yingdi Liu, Hu Liu, Xueying Zeng, Weiguo Wang, Qing Zhang

**Affiliations:** ^1^School of Mathematical Sciences, Ocean University of China, 238 Songling Road, Qingdao, Shandong 266100, China; ^2^School of Computer Science and Technology, Ocean University of China, 238 Songling Road, Qingdao, Shandong 266100, China; ^3^School of Materials Science and Engineering, Ocean University of China, 238 Songling Road, Qingdao, Shandong 266100, China; ^4^Department of Cardiology, Qilu Hospital (Qingdao), Cheeloo College of Medicine, Shandong University, 758 Hefei Road, Qingdao, Shandong 266035, China

## Abstract

Coronary angiography is the “gold standard” for the diagnosis of coronary heart disease, of which vessel segmentation and identification technologies are paid much attention to. However, because of the characteristics of coronary angiograms, such as the complex and variable morphology of coronary artery structure and the noise caused by various factors, there are many difficulties in these studies. To conquer these problems, we design a preprocessing scheme including block-matching and 3D filtering, unsharp masking, contrast-limited adaptive histogram equalization, and multiscale image enhancement to improve the quality of the image and enhance the vascular structure. To achieve vessel segmentation, we use the C-V model to extract the vascular contour. Finally, we propose an improved adaptive tracking algorithm to realize automatic identification of the vascular skeleton. According to our experiments, the vascular structures can be successfully highlighted and the background is restrained by the preprocessing scheme, the continuous contour of the vessel is extracted accurately by the C-V model, and it is verified that the proposed tracking method has higher accuracy and stronger robustness compared with the existing adaptive tracking method.

## 1. Introduction

Cardiovascular disease is currently recognized as one of the most important chronic diseases leading to human death in the world. In recent years, morbidity and mortality from cardiovascular diseases continue to increase, ranking first among various diseases. Coronary angiography (CA) is a common and effective method for diagnosing coronary heart disease. It is regarded as the “gold standard” for the diagnosis of coronary heart disease and is widely used in clinical diagnosis [1].

Normally, human arteries and vessels are invisible under X-rays. However, by injecting X-ray impervious substances into the coronary arteries and then irradiating the coronary artery area with X-rays, the arteries and vessels can be visualized. To decide the treatment plan, doctors need to find the location and degree of coronary artery stenosis based on the image by themselves. Nevertheless, in this way, a large amount of repetitive work and subjective errors are inevitable. Thus, it is of great benefit to invent technologies to segment and identify vessels in angiograms. For this reason, many scholars have proposed various methods.

For many years, image segmentation is one of the focuses of image processing. Up to now, many segmentation technologies for vessels have been proposed. Based on the two characteristics of discontinuity between regions and similarity within regions, we can divide vessel segmentation technologies into three categories: boundary-based segmentation technologies [2–8], region-based segmentation technologies [9–11], and technologies combined with specific theories and tool segmentation [12–15]. Sahoo et al. [16] adopted the maximum entropy method and the gray threshold that maximizes entropy corresponded to the optimal segmentation threshold. Sato et al. [17] constructed a multiparameter similarity function for enhancing vessels by analyzing the properties of the eigenvalues of the Hessian matrix of spherical, tubular, and sheet-like structures at a certain scale. Based on the simplified Mumford-Shah model and the level set idea, Chan and Vese [18] proposed a new active contour C-V model to evolve the curve through the minimization of the energy function. Most recently, deep learning methods have also been widely used in the field of vessel segmentation. For example, Chen et al. [19] trained the 3D U-Net to perform three-dimensional vessel segmentation and achieved high segmentation accuracy.

Moreover, people have studied a variety of methods for vascular identification, such as multiscale-based methods [20–24] and tracking-based methods [25–29]. Among these methods, the tracking-based method has been proved to be very effective. It can detect coronary information based on the local response of angiogram without scanning the entire image. In the process of coronary artery extraction, the extraction result is unstable due to the manual setting of seed points. Aiming at this problem, Xiao et al. [30] proposed an automatic seed point acquisition method based on ridge point detection. These ridge points serve as seed points for adaptive tracking of the centerline of the coronary artery. Aylward and Bullitt [26] proposed a multiscale spatial centerline tracking algorithm based on ridge detection, which uses the eigenvalue decomposition of the Hessian matrix to extract the ridge. However, due to limitations in algorithm design and the effects of low image quality, noise, etc., the accuracy and robustness of these methods still have room for improvement.

Our main work and contributions are as follows: first, we designed a preprocessing scheme to increase the quality of the image and enhance the vascular structure. Then, we used the C-V model to achieve vessel segmentation. Finally, we proposed an improved adaptive tracking algorithm to realize automatic identification of the vascular skeleton, which achieved better effects than former methods according to our experiments.

This paper is organized as follows. In Section 2, we introduce our scheme of image preprocessing.  Section 3 describes the active contour model to extract the vascular contour.  Section 4 describes the details of our proposed improved adaptive tracking method.  Section 5 presents the analysis and experimental results of testing the robustness and accuracy of our methods. Finally, conclusions are drawn in Section 6.

## 2. Image Preprocessing

The complex and varied configuration of the coronary artery structure, noise caused by various factors, artifact caused by the beating of the heart, and low contrast of terminal vessels make precise segmentation very challenging. Therefore, before the extraction of coronary artery structure, coronary angiograms should be preprocessed to enhance the vascular structure and suppress the background noise. In this paper, block-matching and 3D filtering (BM3D) [31] is used to effectively filter out noise. Unsharp masking (UM) [32], contrast-limited adaptive histogram equalization (CLAHE), [33] and multiscale image enhancement [34] are used to improve image contrast and highlight the vascular structure.

### 2.1. Block-Matching and 3D Filtering

BM3D is a 3D block-matching algorithm used primarily for noise reduction in images. Firstly, by the grouping technique of block-matching, image fragments are grouped based on similarity and are integrated into a three-dimensional matrix. Then, filtering is done on every fragment group. At last, the image is transformed back into its two-dimensional form and all overlapping image fragments are weight-averaged to ensure that they are filtered for noise yet retain their distinct signal. This algorithm can effectively remove image noise.

### 2.2. Unsharp Masking

The main procedures of UM algorithm are as follows: first, a passivated fuzzy image is generated after low-pass filtering of the original image. Then, the image with high-frequency components is obtained by subtraction of the original image and the fuzzy image. Finally, the high-frequency image is enlarged with a parameter and superimposed with the original image; that is, an image with enhanced edges is generated. The specific algorithm steps are as follows:

1. Generate the smoothing result:

(1) $$\begin{array}{c} g_{\text{mask}}\left(x,y\right)=I\left(x,y\right)-\overset{-}{I}\left(x,y\right), \end{array}$$

where *I*(*x*, *y*) represents the gray of the pixel (*x*, *y*), $\overset{-}{I}\left(x,y\right)$ represents the gray of the pixel (*x*, *y*) after low-pass filtering, and *g*_mask_(∙) generates the high-frequency component of the image

(2) Add the passivation template to the original image with a certain proportion:

(2) $$\begin{array}{c} \begin{array}{c} \text{g}\left(x,y\right)=I\left(x,y\right)+k*g_{\text{mask}}\left(x,y\right) \end{array}, \end{array}$$

where *k* is the enlarge coefficient and *g*(∙) generates the image with enhanced edges

### 2.3. Contrast-Limited Adaptive Histogram Equalization

As a variant of adaptive histogram equalization, the CLAHE method limits the contrast amplification to reduce excessive amplification of noise. In CLAHE, the contrast amplification in the vicinity of a given pixel is given by the slope of the transformation function, which is proportional to the slope of the neighborhood cumulative distribution function (CDF) and therefore to the value of the histogram. CLAHE limits the amplification by clipping the histogram at a predefined value before computing the CDF. This limits the slope of the CDF and therefore of the transformation function. It is advantageous not to discard the part of the histogram that exceeds the clip limit but to redistribute it equally among all histogram bins. The process of clipping the histogram is shown in Figure 1.

### 2.4. Multiscale Image Enhancement

Frangi et al. [34] proposed the multiscale enhancement method based on the Hessian matrix of the image. In this method, the relationship among the eigenvalues, eigenvectors of the Hessian matrix, and the orientation of vascular structure are utilized, combined with the multiscale theory. Then, the vascular structure in the coronary angiogram is detected by constructing an appropriate vascular similarity function. At present, the method has become one of the most commonly used methods of multiscale enhancement.

The vascular similarity function is established as follows:

(3) $$\begin{array}{c} \begin{array}{c} V\left(P;\sigma \right)=\left\{\begin{array}{c} 0,\text{if }\lambda_{2}>0,\\ \exp\left(-\frac{{R_{B}}^{2}}{2\beta^{2}}\right)\exp\left(-\frac{2{\text{m}}^{2}}{{\lambda_{2}}^{2}}\right)\left(1-\exp\left(-\frac{{S_{H}}^{2}}{2c^{2}}\right)\right),\text{otherwise}, \end{array}\right. \end{array} \end{array}$$

where *λ*_1_ and *λ*_2_ are two eigenvalues of the Hessian matrix, ∣*λ*_1_ | ≤|*λ*_2_|, *P* is an arbitrary point in the image, *σ* is the scale parameter, *R*_*B*_ = |*λ*_1_|/|*λ*_2_|,$\;S_{H}=\sqrt{{\lambda_{1}}^{2}+{\lambda_{2}}^{2}}$, and *R*_*B*_ is the vascular structure enhancement factor, which is used to distinguish the globular structures from the tubular structures; *S*_*H*_ is the norm of the Hessian matrix; and *β*, *c*, and *m* control the overall smoothness of linear objects.

When the scale factor *σ* is consistent with the width of the tubular structure, the filtering result *V*(*P*; *σ*) gets the maximum value. By iterating the scale parameters *σ*, the values *V*(*P*; *σ*) under different scales are obtained, and the maximum value is taken as the actual output of the point *P*:

(4) $$\begin{array}{c} \begin{array}{c} V\left(P\right)=\underset{\sigma_{\min}\leq \sigma \leq \sigma_{\max}}{\max}V\left(P;\sigma \right), \end{array} \end{array}$$

where *σ*_min_ and *σ*_max_ are the minimum and maximum sizes of the vascular structure, respectively.

## 3. Vessel Segmentation

In this section, we will introduce the active contour model to extract the vascular contour of coronary angiograms.

Kass et al. [35] proposed the active contour model (ACM). This method converts the image segmentation problem into solving an energy minimization problem. The contour curve is the edge of the blood vessel when the energy function reaches the minimum. The active contour model is mainly divided into edge-based and region-based according to the different construction methods of the energy function. The most prominent advantage of the ACM is its resistance against strong noise.

The C-V model [18, 36, 37] is a representative region-based active contour model. The specific algorithm steps are as follows:

1. Put forward the energy function:

(5) $$\begin{array}{c} F\left(C,c_{0},c_{b}\right)=u\cdot L\left(C\right)+v\cdot S_{b}\left(C\right)+\lambda_{0}\int_{\text{outside}}\;{\left|I\left(x,y\right)-c_{0}\right|}^{2}dxdy+\lambda_{b}\int_{\text{inside}}\;{\left|I\left(x,y\right)-c_{b}\right|}^{2}dxdy, \end{array}$$

where *c*_0_, *c*_*b*_ represent the average gray levels of the outside and inside areas of the curve *C*, respectively; *L*(*C*) represents the length of the closed curve *C*; *S*_*b*_(*C*) represents the area of the inner area of *C*; and *u*, *v*, *λ*_0_, and *λ*_*b*_ represent the weights of items in the energy function.

(2) Introduce the level set method, set *w*(*x*, *y*) as a sign distance function with positive, negative, zero representing inside, outside, and right on the curve *C*, respectively:

(6) $$\begin{array}{c} \begin{array}{c} \left\{\begin{array}{c} C=\left\{\left(x,y\right)\text{: }w\left(x,y\right)=0\right\},\\ \text{inside}\left(C\right)=\left\{\left(x,y\right)\text{: }w\left(x,y\right)>0\right\},\\ \text{outside}\left(C\right)=\left\{\left(x,y\right)\text{: }w\left(x,y\right)<0\right\}. \end{array}\right. \end{array} \end{array}$$

Introduce the following *H* and *δ* functions:

(7) $$\begin{array}{c} \begin{array}{c} H\left(w\right)=\left\{\begin{array}{c} 1,w\geq 0,\\ 0,w<0, \end{array}\right. \end{array} \end{array}$$

(8) $$\begin{array}{c} \begin{array}{c} \delta \left(w\right)=\frac{d}{dw}H\left(w\right). \end{array} \end{array}$$

Rewrite the energy function as a level set equation:

(9) $$\begin{array}{c} F\left(C,c_{0},c_{b}\right)=u\cdot \int \delta \left(w\right)\left|\nabla w\right|dxdy+v\cdot \int H\left(w\right)dxdy+\lambda_{0}\int_{\text{outside}}\;{\left|I\left(x,y\right)-c_{0}\right|}^{2}\left(1-H\left(w\right)\right)dxdy+\lambda_{b}\int_{\text{inside}}\;{\left|I\left(x,y\right)-c_{b}\right|}^{2}H\left(w\right)dxdy, \end{array}$$

where *λ*_*b*_ and *λ*_0_ are the iterative parameters in the C-V model, and their values affect the evolution rate of the curve *C*. When the curve *C* contains the segmentation target, the internal homogeneity of the curve *C* is low; thus, it is necessary to enlarge *λ*_0_ to accelerate the evolution of the curve *C* to the target, and vice versa.

(3) The energy minimization problem can be solved by minimizing the level set equation iteratively

The C-V model minimizes the energy function to obtain the evolution curve that approaches the edge of the blood vessels and finally segments the target. Compared with other methods, it has better effects on the continuous gradient.

## 4. Improved Adaptive Tracking

In this section, we will propose an improved adaptive tracking method, which is more robust and has fewer misjudgments in the tracking process, to automatically extract the skeleton of the coronary blood vessels.

### 4.1. Ridge Point Detection

Ridge point detection is important for seed point selection, blood vessel tracking, and bifurcation point detection. Ridge point is the local gray maximum point of the two-dimensional image. After multiscale enhancement, a ridge point of the blood vessel is usually located at the maximum point perpendicular to the direction of the blood vessel. The gradient of the local maximum point in the image is zero, and its Hessian matrix is negative [38]. Since the coordinates of image pixels are all integers, according to the principle of linear interpolation, if the point (*ε*, *η*) (*x* < *ε* < *x* + 1, *y* < *η* < *y* + 1) satisfies the following conditions:

(10) $$\begin{array}{c} \begin{array}{c} \nabla \left(x,y\right)\nabla \left(x+1,y+1\right)<0\text{ or}\\ \nabla \left(x+1,y\right)\nabla \left(x,y+1\right)<0,\\ \lambda_{i}\left(x+m,y+n\right)<0,\left(i=1,2,m=0,1,n=0,1\right), \end{array} \end{array}$$

where ∇(*x*, *y*) is the gray gradient of point (*x*, *y*) and *λ*_*i*_(*x*, *y*) are the eigenvalues of the Hessian matrix of point (*x*, *y*); then, (*ε*, *η*) can be considered as a local maximum point, and the pixel (*x*, *y*), as its approximate solution, is defined as a ridge point.

The ridge points may be misjudged due to the image noise caused by the uneven distribution of contrast agents and other factors. Thus, a gray threshold is used to screen out those misjudged ridge points. This method can effectively remove most of the ridge points outside the blood vessel.

### 4.2. Tracking Process

The tracking algorithm starts from a seed point and gradually tracks to the end of the vessel, extracting the blood vessel skeleton. We randomly select the seed point from the detected ridge points.

The initial tracking direction can be calculated from the gray information around the seed point. According to [38], take the seed point as the center and search for the gray maximum point *P*^+^ on the circle with radius *d*. *P*^+^ is the first point of forward tracking, the forward initial tracking direction *u*^+^ and angle *θ*^+^ can be expressed as

(11) $$\begin{array}{c} \;\begin{array}{c} u\left(P^{+}\right)=\frac{P^{+}-P}{||P^{+}-P||}=\left(\cos\theta^{+},\sin\theta^{+}\right). \end{array} \end{array}$$

After obtaining the forward tracking direction, we search for the local maximum point *P*^−^ on arc *l*(2*π* − *θ*^+^ − Δ*θ*, 2*π* − *θ*^+^ + Δ*θ*) centered in the opposite direction (2*π* − *θ*^+^) of the forward tracking angle *θ*^+^. The search area is shown in Figure 2.

The backward direction of the initial trace *u*^−^ can be calculated as

(12) $$\begin{array}{c} \begin{array}{c} u\left(P^{-}\right)=\frac{P^{-}-P}{||P^{-}-P||}. \end{array} \end{array}$$

Tracking from the current point forward to the next point is the main step of this algorithm. The current tracking direction is determined by the direction from the previous point *P*_*k*−1_ to the current point *P*_*k*_:

(13) $$\begin{array}{c} \begin{array}{c} u_{k}=\frac{P_{k-1}-P_{k}}{||P_{k-1}-P_{k}||}. \end{array} \end{array}$$

After determining the tracking direction, we search for the local maximum point *P*_*k*+1_ on arc *l*_*k*_(*θ*_*k*_ − Δ*θ*, *θ*_*k*_ + Δ*θ*) and the following conditions should be met:

(14) $$\begin{array}{c} \begin{array}{c} \left\{\begin{array}{c} I\left(P_{k+1}\right)>I_{0},\\ N_{P}\left(P_{k+1}\right)<\tau_{P}, \end{array}\right. \end{array} \end{array}$$

where *I*(*P*_*k*+1_) is the gray of *P*_*k*+1_, *N*_*P*_(*P*_*k*+1_) is the number of tracking points around *P*_*k*+1_, and *I*_0_ and *τ*_*P*_ are two thresholds. The first condition is to prevent the overtracking beyond the vessel area, while the second condition can avoid repeatedly tracking the vessel and being trapped in a local endless loop. If both conditions are satisfied, we continue to track from *P*_*k*+1_. Otherwise, *P*_*k*+1_ is the endpoint of the vessel. We illustrate the tracking process in Figure 3.

Due to the noise and other issues mentioned above, a few tracking points may deviate from the center of the vessel. The tracking point can be adjusted to the center by center adjustment, which combines the blood vessel contour and tracking direction information. The specific steps are as follows: get the normal line of the vessel through the vertical direction of the current tracking direction and find the intersection points *G*_1_, *G*_2_ of the normal line and the blood vessel contour;, then tracking point *P*_*k*_ can be adjusted to

(15) $$\begin{array}{c} P\prime_{k}=\frac{G_{1}+G_{2}}{2}, \end{array}$$

meanwhile, change the tracking direction *u*_*k*_ to

(16) $$\begin{array}{c} u\prime_{k}=\frac{P\prime_{k}-P_{k-1}}{||P\prime_{k}-P_{k-1}||}. \end{array}$$

The adjustment process is illustrated in Figure 4.

Bifurcation detection is another important process of the tracking algorithm. Ideally, we only need to distinguish two different vessel branches at the vessel bifurcation. However, in the actual tracking process, the accurate positions of vessel bifurcations are usually unknown. Thus, bifurcation detection is required at each point of the tracking process. We propose a robust bifurcation detection method. It includes two main steps: first, obtain one branch point (tracking point) *P*_*k*_ by the tracking method, and second, search in the fan ring area between angle (*θ*_*k*_ − Δ*θ*′,*θ*_*k*_ + Δ*θ*′) and radius (*r*_1_, *r*_2_) to find a ridge point that satisfies the following conditions:

(17) $$\begin{array}{c} \begin{array}{c} \left\{\begin{array}{c} \left|\theta_{b}-\theta_{k}\right|>\tau_{1},\\ \left|\theta_{b}-\theta_{k-1}\right|>\tau_{2},\\ ||P_{b}-P_{k}||>d,\\ N_{B}\left(P_{b}\right)<\tau_{B}, \end{array}\right. \end{array} \end{array}$$

where *P*_*b*_ and *u*(*P*_*b*_) represent the detected ridge point of the new branch (the branch point) and its direction, respectively; *N*_*B*_(*P*_*b*_) is the number of bifurcations around *P*_*b*_; and *τ*_*B*_ is a threshold. The first three conditions mean that when *u*(*P*_*b*_) significantly differs from *u*(*P*_*k*_) and *u*(*P*_*k*−1_) and the distance between *P*_*b*_ and *P*_*k*_ is large enough, the new branch has a large gap with the former branch. The last condition indicates that *N*_*B*_(*P*_*b*_) should be smaller than *τ*_*B*_ to avoid duplication with existing tracking. If all the conditions are satisfied, *P*_*b*_ is detected as a bifurcation point and we keep tracking the branch vessels. The schematic diagram of bifurcation detection is shown in Figure 5.

In addition, before tracking, the ridge image can be preprocessed to remove the scattered and distributed ridge points, it can also reduce the misjudgments of bifurcations. The specific steps areas follows: set a threshold *τ*_*R*_, count the number of surrounding ridge points for each ridge point *N*_*R*_(*P*), and then remove this ridge point if *N*_*R*_(*P*) < *τ*_*R*_ and keep it otherwise.

## 5. Results and Analysis

In this section, we will conduct several experiments to justify the effectiveness of the proposed method. All the images are captured from the video data of coronary angiograms provided by Qilu Hospital (Qingdao). The experiments are implemented on an Intel Core i5-8300H and 8 GB of RAM processor using MATLAB software of version 2019b.

We carefully selected the parameters used. In multiscale enhancement, we set *β*, *c*, and *σ* to 0.5, 20, and [1 : 10]. In the proposed tracking method, we set the radius to 5 pixels and ∆*θ* to 45° in forward tracking. For bifurcation detection, it needs a larger area for searching; thus, we set the radius (*r*_1_, *r*_2_) to (7, 12) pixels and Δ*θ*′ to 135° which can avoid backward tracking. Note that we set other thresholds *I*_0_, *τ*_1_, *τ*_2_, *d*, *τ*_*P*_, *τ*_*B*_, and *τ*_*R*_ to 10, 45°, 30°, 5, 4, 2, and 3.

Three images with the different vascular structures were selected for independent experiments, which are shown in Figure 6. We applied our methods for these images, and the results are shown in Figure 7.

As can be seen from Figure 7, even though the vascular structures in the images are very different, the proposed method still has a nice experimental effect. From the images preprocessed (a), we can find that after the image preprocessing, the vascular structures were successfully highlighted and the background was restrained. The extraction of vessel contours (b) obtained vascular contours accurately and completely. The improved adaptive tracking method (c) is a core part of our work: compared with the original adaptive tracking method of [38], one of the main improvements in this approach is the bifurcation point detection part. We changed the originally fixed search radius to a proper search scope, which enhanced the capacity of the retrieval of bifurcation, and we used four conditions in Equation (17) to judge bifurcation point instead of only using the first condition, which greatly improved the detection accuracy and reduced the misjudgment. The results can be seen in Figure 8.

To achieve the completely automatic identification of vessels, we need to test the robustness of the proposed tracking method for randomly selected seed points from the detected ridge points. Taking Figure 6(c) as an example, three seed points were selected from different positions. The experimental results are shown in Figure 9. It can be seen that the results of the proposed method have strong robustness; that is, our method is generally applicable for automatically selected seed points. Meanwhile, our method is more accurate than the method of [38], which is clear in Figure 9 that the points of different types we identified are more approaching to the real vessel.

Even though our method has an improvement in accuracy and robustness compared to the former one, it still has some shortcomings. For example, the image preprocessing method is not effective enough for some images with complex vascular structures. Although the detection of bifurcation points has been improved compared with the method in [38], there are still a few misjudgments. This phenomenon can be seen in Figure 8(b). In the case of a more complex vascular structure, the tracking effect varies with the selection of seed points, and some vessel segments may be lost, as shown in Figure 7(c2).

## 6. Conclusion

In this paper, we designed a scheme of image preprocessing, used the C-V model, and proposed an improved adaptive tracking method, with which we can realize segmentation and automatic identification of vessels in coronary angiograms. Among these methods, the improved adaptive tracking method contains our major innovations that can enhance the capability of identifying vessels. Besides, we did many experiments to test our proposed method and the results turned out that our method is more robust and accurate than the former method.

Due to the complexity of coronary angiograms described above, traditional image processing methods are not effective enough. Hence, in the following work, we will continue to optimize the tracking algorithm and carry out image process research on deep learning to achieve a better effect.

## Figures and Tables

**Figure 1:** The clipping process of CLAHE.

**Figure 2:** Initial direction detection.

**Figure 3:** Forward tracking.

**Figure 4:** Centerline adjustment.

**Figure 5:** Vascular branch detection.

**Figure 6:** Three selected original images.

**Figure 7:** Experimental results of three original images obtained by applying the proposed method. (a) Images preprocessed. (b) Vascular contour segmentation. (c) Improved adaptive tracking (red dots are bifurcation points, green dots are normal tracking points).

**Figure 8:** Comparison of the tracking effect between our proposed method and the method of [38]. (a) Results of [38]. (b) Results of the proposed method.

**Figure 9:** Experimental results of different seed points (blue). (a) The method of [38]. (b) The proposed method.

## Data Availability

The data supporting this study is from Qilu Hospital (Qingdao) of Shandong University.
